The article "Impact of Systematic Holistic Nursing Combined with Narrative Nursing Intervention for Patients with Advanced Gastric Cancer on Complications and Negative Emotions" was retracted in 2023. Reasons: signs of a paper mill; compromised peer review; unreliable results or conclusions.

# Impact of Systematic Holistic Nursing Combined with Narrative Nursing Intervention for Patients with Advanced Gastric Cancer on Complications and Negative Emotions

**DOI:** 10.1155/2022/9148843

**Published:** 2022-07-15

**Authors:** Hui Lu, Lingyun Zhu, Chunxiao Tan

**Affiliations:** ^1^Department of Gastroenterology, Affiliated Hospital of Jiangnan University, Wuxi, Jiangsu 214000, China; ^2^Department of Gastroenterology, Affiliated Wuxi 2 People's Hospital of Nanjing Medical University, Wuxi, Jiangsu 214000, China

## Abstract

**Objective:**

The aim of this study is to evaluate the influence of systemic holistic nursing combined with narrative nursing on the postoperative complications and negative emotions in patients with advanced gastric cancer.

**Methods:**

A total of 120 patients with advanced gastric cancer admitted to our hospital between February 2020 and February 2021 were recruited and assigned to receive systemic holistic nursing combined with narrative nursing (experimental group) or systemic holistic nursing (control group) according to order of admission, with 60 cases in each group. The outcome measures included the incidence of postoperative complications, negative emotion score, quality of life score, self-efficacy score, self-care ability score, and nursing satisfaction.

**Results:**

The experimental group had a significantly lower incidence of complications and lower negative emotion scores than the control group (*P* < 0.001). Systemic holistic nursing plus narrative nursing resulted in significantly higher life scores, self-efficacy scores, and self-care ability scores in the experimental group after nursing than in the control group (*P* < 0.001). Patients of the experimental groups were more satisfied with the nursing in contrast to those in the control group (*P* < 0.001).

**Conclusion:**

Systematic holistic nursing plus narrative nursing alleviates the negative emotions of patients, improves their self-efficacy scores, lowers the incidence of complications, and enhances quality of life.

## 1. Introduction

Gastric cancer is a common malignant tumor, with its incidence ranking first among gastrointestinal malignancies. The Cancer development is promoted by both genetic and environmental factors, and around 50% of cancer is provoked by environmental agents. The disease is not prevalent in the young population (under 45 years of age), with a prevalence of about 10%. Clinically, surgery and chemotherapy are the mainstays for treatment. However, surgery may trigger complications such as anastomotic fistula, lung infection, gastrointestinal dysfunction, and chemotherapy may result in liver, kidney, and other organ damage, critically hindering the quality of life of patients [1–3]. The middle-aged and elderly population are more susceptible to gastric cancer [4], and it has mostly developed to an the advanced stage at the time of diagnosis due to the insidiousness of early symptoms [5]. In addition to serious clinical stress responses, patients may also be subjected to obvious negative emotions and even depression and anxiety in severe cases [6, 7], which further undermines the efficacy of surgery and chemotherapy. Moreover, systemic chemotherapy outcomes are dismal, with a median survival of 6–11 months. To improve the clinical efficacy of patients with advanced gastric cancer and relieve their physical and psychological stress, comprehensive nursing is frequently applied in clinical practice for perioperative care, which lowers the incidence of postoperative complications but fails to alleviate patients' psychological stress. Thus, it is of great significance to explore high-quality nursing models centered on psychological intervention.

The article "Impact of Systematic Holistic Nursing Combined with Narrative Nursing Intervention for Patients with Advanced Gastric Cancer on Complications and Negative Emotions" was retracted in 2023. Reasons: signs of a paper mill; compromised peer review; unreliable results or conclusions.

Systematic holistic nursing is the systematization and integration of comprehensive nursing interventions, which eliminates the triviality of traditional nursing and makes clinical nursing more scientific. Holistic nursing covers an aspect of the overall experience, both physically and emotionally, of the response and effects of the disease on the individuals and families. Moreover, this nursing model is carried out to mitigate the negative emotions of patients with a strong targeted effect. A prior study has revealed that systematic holistic nursing could improve cancer-related fatigue in cases with advanced gastric cancer undergoing chemotherapy [8]. However, its impact on postoperative complications is still unclear. Currently, as the psychological care in systemic holistic nursing is still confined to the shackles of conventional nursing, whether the introduction of more advanced psychological nursing can further enhance the effect of systemic holistic nursing remains elusive. Accordingly, narrative nursing is incorporated in this study. In narrative nursing, nurses help patients develop a positive life attitude and regain their self-value by storytelling to share the essence of nursing.

The results of the application of systematic holistic nursing specific intervention results for patients with advanced gastric cancer are as follows.

## 2. Materials and Methods

### 2.1. General Information

The medical data of 120 patients with advanced gastric cancer admitted to our hospital between February 2020 and February 2021 were retrospectively analyzed.

Inclusion criteria: patients who were diagnosed with gastric cancer by tumor marker detection and pathological examination [9], with the TNM staging of stage III or IV, who met the indications for gastric cancer surgery [7], with stable vital signs after the surgery, without a history of other tumors, with a Karnofsky score of >60 points [10], and who had a detailed understanding of the main objectives of the study and the specific implementation needs of the study and provided written informed consent were included.

The article "Impact of Systematic Holistic Nursing Combined with Narrative Nursing Intervention for Patients with Advanced Gastric Cancer on Complications and Negative Emotions" was retracted in 2023. Reasons: signs of a paper mill; compromised peer review; unreliable results or conclusions.

Exclusion criteria: patients with mental problems that prevent communication, with other malignant tumors, abnormal blood systems, liver, kidney, heart, brain, and other organ disorders, with contraindications to surgery [11] were excluded. All 120 cases were enrolled and divided into the experimental group (*n* = 60) and the control group (*n* = 60). The two groups presented no significant difference in baseline data (*P* > 0.05, Table 1). The study was ratified by the ethics committee.

### 2.2. Withdrawal Criteria

(1) Patients with adverse events or serious adverse events; (2) with deterioration during the experiment; (3) with complications; and (4) who were unwilling to participate in the subsequent clinical trial and provoked their consent were excluded.

## 3. Method

All cases were given systematic holistic nursing, the specific steps were as follows: (1) *Nursing protocol formulation.* After enrollment, the clinical data of the patients were analyzed in detail to evaluate their psychological status. Nursing protocols were formulated according to the patients' actual situation, including general nursing, psychological nursing, and health education. The patients' conditions and feedback were recorded promptly for further adjustment of the nursing plans. (2) *Health education*. Different groups were divided based on the patients' education level and religious beliefs. Health education manuals of advanced cancers were distributed to all patients, and the key contents were explained to patients and their families. Chief physicians, nutritionists, and psychologists were invited to give health education lectures regularly. (3) *General nursing*. The cleanliness of the ward, visiting time, and the number of visitors was under strict control to avoid cross-infection. The patients were instructed to perform deep breathing exercises and were assisted in gesture changing and expectoration through manual tremor and atomization inhalation. The drainage tubes were secured and prevented from distortion or obstruction. The drainage fluid was closely monitored, and any abnormalities were reported immediately. The surgical wounds were kept dry to prevent pressure sores. The nursing staff administered medicines to patients according to the doctor's advice, observed changes in patients' physical signs, and strengthened gastrointestinal decompression nursing. (4) *Dietary nursing*. The large amount of ascites in patients resulted in a poor appetite and a risk of malnutrition. Dietary instructions were given according to the patient's eating habits, including a high-calorie and high-protein diet, a daylong stream of mini-meals, and a light diet for patients with severe gastrointestinal reactions. Appropriate antiemetic drugs were given if necessary. (5) *Sports nursing*. The patients were assisted to turn over 2 hours after the operation, sit up after 1 day, perform bedside exercise after 2 days, and exercise indoors after 3 days. (6) *Psychological nursing.* The nursing staff communicated with patients every week to help eliminate their negative emotions and provide more psychological support.

The article "Impact of Systematic Holistic Nursing Combined with Narrative Nursing Intervention for Patients with Advanced Gastric Cancer on Complications and Negative Emotions" was retracted in 2023. Reasons: signs of a paper mill; compromised peer review; unreliable results or conclusions.

The experimental group additionally received a narrative nursing intervention. The specific steps were as follows: (1) The nursing staff received training from psychologists, to master psychological nursing skills and ensure the professionality and scientificity of the nursing. (2) The nursing staff communicated with patients face-to-face every day and guided the patients to share their stories and daily issues, assess the impact of the problems, and explore the reasons and appropriate solutions in daily nursing. (3) Personalized nursing programs were developed to enhance daily communication with the patients and understand their psychological needs. The patients were instructed to examine their situations and problems more objectively to further alleviate their psychological pressure. (4) The nursing staff communicated with the patients' family members to provide family support for the patients and enhance their positive outlook on life.

### 3.1. Observational Criteria

1. Complication rate: complications include pulmonary infection, atelectasis, incision infection, anastomotic fistula, gastric dysfunction, and pressure ulcers.
2. Negative emotion score: emotional state of the patients between nursing was evaluated based on the hospital anxiety and depression (HAD) Scale [12]. The HADS-A includes 7 items that assess generalized anxiety including tension, worry, fear, panic, difficulties in relaxing, and restlessness. Responses are rated on a 4-point Likert scale and range from 0 to 3.
3. Quality of life score: generic Quality of Life Inventory-74 Scale (GQOLI-74) [13] was used to assess the quality of life of all groups of patients between nursing. The scale contains four scoring factors: mental function, physical function, social function, and material life status, all score of 100 points. The higher the score, the better the level of life of the patients.
4. Self-efficacy score: self-efficacy scores of all cases between the nursing were evaluated according to the general self-efficacy scale (GSES) [14]. The GSES is a self-reported measure that includes 10 questions scored on a 4-point Likert scale; the total score is the sum of all items evaluated. Scores on this scale range between 10 and 40, with a higher score indicating greater self-efficacy.
5. Self-care ability score: the hospital's self-developed questionnaire was used to investigate the patient's mastery of advanced gastric cancer health knowledge and home care skills before and after nursing. The scores for each item are between 0–100 points. A higher score indicates better patients' self-care ability.
6. Nursing satisfaction: the hospital's self-developed scale was used to assess the patients' nursing satisfaction. The scoring range is between 0–5 stars, with 5 stars being highly satisfied, 3 and 4 stars being satisfied, and below being dissatisfied.

The article "Impact of Systematic Holistic Nursing Combined with Narrative Nursing Intervention for Patients with Advanced Gastric Cancer on Complications and Negative Emotions" was retracted in 2023. Reasons: signs of a paper mill; compromised peer review; unreliable results or conclusions.

### 3.2. Statistical Method

In this study, SPSS20.0 was used for statistical processing. Graphpad Prism 7 software was used to plot the graphics. Research includes counting data and measurement data. Counting data were analyzed using the chi-square test and the measurement data were analyzed using the *t*-test. *P* > 0.05 was used as a cut-off value for statistical significance.

## 4. Results

### 4.1. Complication

The incidence of complications in the experimental group was significantly lower than that of the control group (*P* < 0.001), as shown in Figure 1.

### 4.2. Negative Emotion Scores

After nursing, lower negative emotion scores were observed in the experimental group (*P* < 0.001) (Figure 2).

### 4.3. Quality of Life Scores

The experimental group had higher quality of life scores than the control group (*P* < 0.001), as shown in Figure 3.

### 4.4. Self-Efficacy Scores

Self-efficacy scores of the experimental group after nursing were remarkably higher than those of the control group (*P* < 0.001) (Figure 4).

### 4.5. Self-Care Ability Scores

The experimental group had higher self-care ability scores than the control group (*P* < 0.001) (Table 2).

### 4.6. Nursing Satisfaction

Patients in the experimental group were more satisfied with the nursing (*P* < 0.05) (Table 3).

## 5. Discussion

Gastric cancer is a malignant tumor originating from the gastric mucosal epithelium with hidden symptoms in the early stages. Most cases are at the advanced stages of disease at the time of diagnosis, during which surgery and chemotherapy are the main treatment methods [15]. As advanced-stage malignant tumors are serious stressors [16], invasive treatment methods such as surgery may result in negative emotions in patients such as anxiety, depression, and fear [17], seriously compromising the treatment effect and quality of life of patients. To improve the psychological state of cases and enhance the influence of surgery, comprehensive nursing is frequently applied for intervention in clinical scenarios; nonetheless, previous research revealed that comprehensive nursing intervention failed to alleviate the negative emotions of patients [18], which highlights the importance of a more targeted nursing model for patients with advanced gastric cancer. The systematic holistic nursing intervention used in the present study is a high-quality nursing model with psychological nursing as the core that integrates health education, general nursing, and dietary guidance during nursing. It monitors the patient's condition changes in real-time and adjusts the nursing scheme promptly according to the patient's feedback. Previous research has applied systemic holistic nursing in the nursing of patients with advanced gastric cancer after chemotherapy and found that cancer-related fatigue after treatment was significantly reduced and their quality of life has been significantly improved [19].

The article "Impact of Systematic Holistic Nursing Combined with Narrative Nursing Intervention for Patients with Advanced Gastric Cancer on Complications and Negative Emotions" was retracted in 2023. Reasons: signs of a paper mill; compromised peer review; unreliable results or conclusions.

However, the application of systemic holistic nursing intervention shows no major breakthrough in terms of psychological nursing when compared with conventional psychological nursing. Accordingly, narrative nursing was employed in addition to systematic holistic nursing in the present study. Specifically, the psychological care in the systematic holistic nursing intervention is replaced with more scientific and advanced narrative nursing that helps patients abandon bad lifestyles and establishes a positive life attitude through storytelling. Anja et al. stated that the essence of narrative nursing is to absorb and accept patients' stories and assist them to reconstruct the meaning of life, thereby achieving the purpose of psychological care [20]. The study showed lower negative emotion scores in the experimental group after nursing (*P* < 0.001), and patients in the experimental group had a stronger sense of self-efficacy, suggesting that narrative medicine fully alleviated the negative emotions of patients and enhanced their psychological health.

In addition to patients, narrative medicine also has a positive effect on patients' families. It contributes to maintaining and enhancing communication between the patients and their families, which mitigates the negative psychological conditions of the family members. Thronicke A et al. revealed that narrative nursing provides hope for the patients' families in terms of the patients' condition, which leads to better family care and positive family support [21]. There are potential limitations to this study. Firstly, this study did not include objective measurements of nursing satisfaction, so the reported nursing satisfaction in this study is subjected to reporting biases. Secondly, this study was conducted on a relatively homogenous population, so the generalizability of these findings may be limited to similar disease backgrounds. Thirdly, the sample size was relatively small. Hence, ongoing studies are warranted to overcome these problems.

The article "Impact of Systematic Holistic Nursing Combined with Narrative Nursing Intervention for Patients with Advanced Gastric Cancer on Complications and Negative Emotions" was retracted in 2023. Reasons: signs of a paper mill; compromised peer review; unreliable results or conclusions.

In conclusion, systematic holistic nursing combined with narrative nursing effectively alleviates the negative emotions of patients with advanced gastric cancer, improves their self-efficacy and self-care ability, lowers the incidence of complications, and ensures a good quality of life [8, 22, 23].

## Figures and Tables

**Figure 1:** Comparison of the incidence of complications between the two groups of patients (n (%)). Note: Figure 1(a) is the experimental group, and Figure 1(b) is the control group. In the figure, the black area is lung infection, the dark gray area is atelectasis, the light gray area is incision infection, the white area is an anastomotic fistula, the black grid area is gastric dysfunction, the dark gray grid area is pressure ulcer, and the light gray grid area is no complication. # indicates *P* < 0.001. There were no significant differences in the incidence of lung infection, atelectasis, incision infection, anastomotic fistula, gastric dysfunction, and pressure ulcer between the two groups (2 vs 4, 1 vs 5, 1 vs 6, 2 vs 6, 1 vs 6, 0 vs 5, *P* > 0.05). More patients had no complications in the experimental group than the control group (53 vs 28, *P* < 0.001).

**Figure 2:** Comparison of negative emotion scores of the two groups of patients (*x̅* ± *s*, points). Note: Figure 2(a) is the HAD-A score, and Figure 2(b) is the HAD-D score; the abscissas of the two figures from left to right are before and after nursing; the dotted line in the figure is the experimental group, and the square line is the control group; # indicates *P* > 0.05. The HAD-A score and HAD-D score before nursing between the experimental group and the control group were not statistically different (8.10 ± 1.00 vs 8.13 ± 1.01, 7.98 ± 1.20 vs 7.96 ± 1.12, *P* > 0.05); the HAD-A and HAD-D scores of the experimental group after nursing were significantly lower than those of the control group (5.15 ± 0.98 vs 6.24 ± 0.98, 5.10 ± 0.87 vs 6.19 ± 0.86, *P* < 0.001).

**Figure 3:** Comparison of quality of life scores between the two groups of patients (*x̅* ± *s*, points). Note: the abscissas of Figures 3(a) and 3(b) represent psychological function, physical function, social function, and material life status from left to right. The black area in the figure is the experimental group, and the gray area is the control group; # indicates *P* < 0.001. Figure 3(a) shows the quality of life score before nursing. There was no statistical difference in the scores of psychological function, physical function, social function, and material life state between the two groups before nursing (49.26 ± 5.21 vs 49.32 ± 5.20, 60.26 ± 5.21 vs 60.23 ± 5.12, 49.88 ± 5.32 vs 49.78 ± 5.20, 46.52 ± 4.52 vs 46.58 ± 4.20, *P* > 0.05). Figure 3(b) shows the quality of life score after nursing. The scores of mental function, physical function, social function, and material life state of the experimental group after nursing were significantly higher than those of the control group (62.15 ± 3.58 vs 54.26 ± 4.10, 70.89 ± 3.68 vs 62.98 ± 3.89, 60.23 ± 4.20 vs 52.98 ± 3.65, 62.11 ± 3.65 vs 52.53 ± 4.14, *P* < 0.001).

The article "Impact of Systematic Holistic Nursing Combined with Narrative Nursing Intervention for Patients with Advanced Gastric Cancer on Complications and Negative Emotions" was retracted in 2023. Reasons: signs of a paper mill; compromised peer review; unreliable results or conclusions.

**Figure 4:** Comparison of self-efficacy scores between the two groups of patients (*x̅* ± *s*, points). Note: in Figure 4, the abscissa is from left to right before and after nursing, and the ordinate is the self-efficacy score (points); the black area in the figure is the experimental group, and the gray area is the control group; # indicates *P* < 0.001. There was no statistical difference in the self-efficacy scores of the two groups before nursing (20.13 ± 2.65 vs 20.15 ± 2.68, *P* > 0.05); the self-efficacy scores of the experimental group after nursing were significantly higher than those of the control group (30.12 ± 2.45 vs 24.68 ± 2.68, *P* < 0.001).

**Table 1:** Comparison of general information of patients.

Groups	Experimental group (*n* = 60)	Control group (*n* = 60)	X^2^/*t*	*P*
Gender			0.037	0.847
Male	39	40		
Female	21	20		

Age (years)				
Range	45–76	46–74		
Average age	60.23 ± 2.10	60.45 ± 2.12	0.571	0.569
Average weight (kg)	53.26 ± 2.50	53.68 ± 2.10	0.996	0.321
BMI (kg/m^2^)	20.42 ± 2.15	20.52 ± 2.23	0.250	0.803

TNM staging			0.139	0.709
III	35	37		
IV	25	23		
Karnofsky score	65.22 ± 2.10	64.98 ± 2.15	0.619	0.537

Pathological classification				
Adenocarcinoma	38	36	0.141	0.707
Signet-ring cell carcinoma	18	18	0.000	1.000
Small cell lung carcinoma	4	6	0.436	0.509

Underlying disease				
Diabetes	12	11	0.054	0.817
Hypertension	16	18	0.164	0.685
Lung disease	10	9	0.063	0.803

Lesion				
Gastric cardia cancer	20	21	0.037	0.847
Gastric cancer invading cardia	30	30	0.000	1.000
Total gastric cancer	1	2	0.342	0.559
Remnant gastric cancer	9	7	0.289	0.591

Education level			0.034	0.853
High school and below	25	26		
University and above	35	34		

The article "Impact of Systematic Holistic Nursing Combined with Narrative Nursing Intervention for Patients with Advanced Gastric Cancer on Complications and Negative Emotions" was retracted in 2023. Reasons: signs of a paper mill; compromised peer review; unreliable results or conclusions.

**Table 2:** Comparison of self-care ability scores between the two groups (*x̅* ± *s*, points).

Items	Experimental group		Control group		*t*	*P*
Mastery of gastric cancer knowledge	Before nursing	40.26 ± 2.65	Before nursing	40.37 ± 2.56	0.231	0.818
	After nursing	89.98 ± 5.40	After nursing	79.21 ± 5.22	11.108	<0.001
	*t*	64.026	*t*	51.747		
	*P*	<0.001	*P*	<0.001		
Mastery of home nursing skills	Before nursing	46.98 ± 2.58	Before nursing	47.00 ± 2.10	0.047	0.963
	After nursing	92.35 ± 2.54	After nursing	85.26 ± 3.54	12.605	<0.001
	*t*	97.068	*t*	72.002		
	*P*	<0.001	*P*	<0.001		

**Table 3:** Comparison of nursing satisfaction between the two groups of patients [n(%)].

Groups	*n*	Very satisfied	Satisfied	Dissatisfied	Total satisfaction
Experimental group	60	24 (40.0)	34 (56.7)	2 (3.3)	58 (96.7)
Control group	60	18 (30.0)	32 (53.3)	10 (16.7)	50 (83.3)
**X** ^**2**^		1.319	0.135	5.926	5.926
***P***		0.251	0.714	0.015	0.015

## Data Availability

No data were used to support this study.
